# Bayesian Gene Selection Based on Pathway Information and Network-Constrained Regularization

**DOI:** 10.1155/2021/7471516

**Published:** 2021-08-04

**Authors:** Ming Cao, Yue Fan, Qinke Peng

**Affiliations:** ^1^Faculty of Electronic and Information Engineering, Xi'an Jiaotong University, Xi'an 710049, China; ^2^School of Mathematics and Statistics, Shaanxi Xueqian Normal University, Xi'an 710100, China

## Abstract

High-throughput data make it possible to study expression levels of thousands of genes simultaneously under a particular condition. However, only few of the genes are discriminatively expressed. How to identify these biomarkers precisely is significant for disease diagnosis, prognosis, and therapy. Many studies utilized pathway information to identify the biomarkers. However, most of these studies only incorporate the group information while the pathway structural information is ignored. In this paper, we proposed a Bayesian gene selection with a network-constrained regularization method, which can incorporate the pathway structural information as priors to perform gene selection. All the priors are conjugated; thus, the parameters can be estimated effectively through Gibbs sampling. We present the application of our method on 6 microarray datasets, comparing with Bayesian Lasso, Bayesian Elastic Net, and Bayesian Fused Lasso. The results show that our method performs better than other Bayesian methods and pathway structural information can improve the result.

## 1. Introduction

Identifying disease-associated genes, which can be treated as diagnostic biomarkers, can bring a significant effect on disease diagnosis, prognosis, and treatments [1, 2]. With the development of high-throughput technologies in recent years, gene expression profiling has provided a useful way to find biomarkers. Researchers can identify the genes which are differentially expressed between two groups of samples. These genes are regarded as disease-associated genes. However, gene expression data usually contains a large number of genes and a relatively small sample size [3, 4]. And many of the genes are also redundant or irrelevant to the prediction [5, 6]. Furthermore, there are also noises in the experiment procedures which will influence the gene expression values. Therefore, identifying the biomarkers from gene expression data is challenging.

During the last decades, a number of gene selection methods have been developed to tackle this problem. Feature selection and feature extraction are two major methods (we treat gene and feature equally in this paper). On the one hand, the aim of feature selection is to select relevant features and do not change the form of the features. On the other hand, feature extraction will extract the feature from the original data and may alter the form of the features. Here, we focus on the feature selection methods since the results of such methods could be interpreted easily. Feature selection methods can be generally organized into three categories: filter, wrapper, and embedded methods. Both the wrapper and embedded methods are classifier-dependent methods; thus, they are always time consuming and easy to overfitting. However, the filter methods are usually based on statistic approaches [7] such as mRMR [5], PLSRFE [8], lasso [9], and elastic net [10], which are relatively efficient in terms of computation and can derive a score of each of the genes which represents the significance of the gene. Therefore, we focus on the filter methods in this paper.

Although these methods are successful in many applications, they usually obtain suboptimal solutions. Therefore, the prediction accuracies are not satisfied and the disease-associated genes selected from different methods have few overlaps [11]. This is partly due to the fact that the discriminatory power of many biomarkers is similar. Furthermore, some genes which have low discriminatory powers play important roles in cellular functions. Their combinations are highly discriminative while they are usually ignored [12, 13].

Recently, with a large amount of biological information accumulated, there is an increased interest in gene selection with incorporating information on pathways, which can partially compensate for the lack of reliable expression data [14]. Pathways depict a series of chemical interactions in living cells; genes that interact with one another usually mean that they function together concertedly. Therefore, these genes should be highly correlated and have dependence structures. However, many studies only utilize the information that pathways cluster genes into the natural group; the pathway structural information is neglected. Li and Li have overcome this disadvantage by incorporating pathway structure information through a Laplacian matrix of a global graph [15, 16] and combined with lasso penalty to perform network-constrained penalty which can select subgroups of correlated features in the network. This penalty is based on the assumption that genes belonging to the same pathway have similar functions and therefore smoothed regression coefficients. And this penalty has been successfully applied in many studies [17–19].

The Bayesian approach has three major advantages over Bayesian selection methods [20]. Firstly, hyperparameters can be estimated automatically through fulfilling stochastic draws; thus, 10-fold cross-validation for estimating penalized parameters is not required. Secondly, the Bayesian framework can utilize the pathway information naturally by integrating it in the model as prior knowledge. Finally, the Bayesian estimation with the posterior distributions can provide credible intervals for the regression coefficients, which is a great advantage over frequentist methods.

In this paper, we work with a Bayesian framework to perform gene selection through network-constrained regularization. Similar to the Bayesian Lasso [21], Bayesian Elastic Net [22], and Bayesian Fused Lasso [23], we use shrinkage priors to perform regularization. We show that all the conditional posteriors of the proposed model are available in closed form and proper. Thus, parameter estimation can be performed through Gibbs sampling easily. The pathway information is obtained from the Kyoto Encyclopedia of Genes and Genomes (KEGG) [24], which is the most popular pathway public database, especially pathways associated with several types of cancer could be obtained in the model. Furthermore, following Held and Holmes [25], we extend the regression model to binary regression which can perform binary classification through an auxiliary variable. This method is assessed by applying it to several microarray datasets.

## 2. Method

### 2.1. The Bayesian Network-Constrained Model for Gene Selection

Considering an *N* × *P* matrix *X*, where *P* is the number of genes and *N* is the number of the samples, with a response vector *y* = (*y*_1_, ⋯,*y*_*n*_)^*T*^, we normalize the values of each feature as the tradition in variable selection; thus, the mean and standard deviation of each feature are 0 and 1. We assume the likelihood function of the continuous response is Gaussian function:

(1) $$\begin{array}{c} Y\;|\;X,\beta ,\sigma^{2}∼N_{n}\left(X\beta ,\sigma^{2}I_{n}\right), \end{array}$$

which can be also expressed as

(2) $$\begin{array}{c} y=X\beta +\varepsilon ,\varepsilon ∼N_{n}\left(0,\sigma^{2}I_{n}\right). \end{array}$$

Following Li and Li's work [16], we incorporate the pathway information through its normalized Laplacian matrix. Consider an undirected graph *G* = (*V*, *E*, *W*). In this graph, genes are represented by a set of nodes *V*, and the interactions between genes are represented by a set of edges *E* = {*u* ~ *v*}, and *W* is the weights of the edges, where *w*(*u*, *v*) represents the weight of edge *e* = (*u* ~ *v*) which indicates the uncertainty of the edge between the vertices *u* and *v*. The degree of each vertex is defined as *d*_*v*_ = ∑_*u*∼*v*_*w*(*u*, *v*). Then, the normalized Laplacian matrix *L* for graph *G* with the *u*th and *v*th elements can be defined by

(3) $$\begin{array}{c} L\left(u,v\right)=\left\{\begin{array}{c} 1-\frac{w\left(u,v\right)}{d_{u}},\;\text{if }u=v\text{ and }d_{u}\neq 0,\\ -\frac{w\left(u,v\right)}{\sqrt{d_{u}d_{v}}},\;\text{if }u\text{ and }v\text{ are adjacent},\\ 0,\text{otherwise}. \end{array}\right. \end{array}$$

Here, we let *w*(*u*, *v*) = 1 if there exists an interaction between gene *u* and *v*, and *w*(*u*, *v*) = 0, otherwise.

To form the network-constrained regularization, we assign the prior distribution for *β* as follows:

(4) $$\begin{array}{c} \beta ∼N_{p}\left(0,\frac{\sigma^{2}}{r}\Lambda^{-1}\right), \end{array}$$

where *Λ* is taking the form:

(5) $$\begin{array}{c} \Lambda =\mathrm{diag}\left(\tau_{1}^{-1},\tau_{2}^{-1},\cdots ,\tau_{p}^{-1}\right)+L=\left\{\begin{array}{cccc} 1+\tau_{1}^{-1} & L\left(1,2\right) & \cdots & L\left(1,p\right)\\ L\left(2,1\right) & 1+\tau_{2}^{-1} & \cdots & L\left(2,p\right)\\ \vdots & \vdots & \ddots & \vdots \\ L\left(p,1\right) & L\left(p,2\right) & \cdots & 1+\tau_{p}^{-1} \end{array}\right\}. \end{array}$$

Note that *Λ* only contains hyperparameter *τ*.

To eliminate the |*Λ*|^1/2^ in the prior distribution of *β*, we assign the prior distribution for *τ* as follows:

(6) $$\begin{array}{c} p\left(\tau^{2}\;|\;\lambda \right)=C_{\tau }{\left|\Lambda \right|}^{-1/2}\overset{p}{\underset{j=1}{\prod }}\frac{\lambda^{2}}{2}\exp\left(-\frac{\lambda^{2}}{2}\tau_{j}^{2}\right), \end{array}$$

where *C*_*τ*_ is the normalizing constant.

The prior distribution defined in (6) is proper, due to the following analysis:

Let *A* = *Λ* − *I*_*n*_, and *A* is a symmetric and positive semidefinite matrix.

Let *D*_*A*_ = diag(*a*_1_, ⋯, *a*_*p*_), where *a*_1_, ⋯, *a*_*p*_ are eigenvalues of *A* and 0 ≤ *a*_1_ ≤ ⋯≤*a*_*p*_.

Since *A* is the symmetric and positive semidefinite, there exists an orthonormal matrix *Q*. Hence, the eigendecomposition of matrix *A* can be written as *A* = *QD*_*A*_*Q*^*T*^.

Because of *Λ* = *A* + *I*_*n*_ = *QD*_*A*_*Q*^*T*^ + *QQ*^*T*^ = *Q*(*D*_*A*_ + *I*_*n*_)*Q*^*T*^, so ∣*Λ* | = ∏_*i*=1_^*n*^(*a*_*i*_ + 1) ≥ 1.

Then,

(7) $$\begin{array}{c} \int_{0}^{\infty }C_{\tau }{\left|\Lambda \right|}^{-1/2}\overset{p}{\underset{j=1}{\prod }}\frac{\lambda^{2}}{2}\exp\left(-\frac{\lambda^{2}}{2}\tau_{j}^{2}\right)d\tau^{2}\leq C_{\tau }\int_{0}^{\infty }\overset{p}{\underset{j=1}{\prod }}\frac{\lambda^{2}}{2}\exp\left(-\frac{\lambda^{2}}{2}\tau_{j}^{2}\right)d\tau^{2}<\infty , \end{array}$$

where the integrand is kernels of the gamma density that indicates the integral is finite. Therefore, the prior distribution is proper.

Since

(8) $$\begin{array}{c} \beta^{T}\Lambda \beta =\beta^{T}D^{-1}\beta +\underset{u∼v}{\sum }{\left(\frac{\beta_{u}}{\sqrt{d_{u}}}-\frac{\beta_{v}}{\sqrt{d_{v}}}\right)}^{2}\geq 0,\;D=\mathrm{diag}\left(\tau_{1}^{2},\tau_{2}^{2},\cdots ,\tau_{p}^{2}\right), \end{array}$$

*Λ* is positive semidefinite.

The joint posterior distribution can be written as

(9) $$\begin{array}{c} p\left(\beta ,\lambda ,\sigma^{2},\tau^{2},r\;|\;X,Y\right)\propto {\left(\sigma^{2}\right)}^{-n/2}\exp\left(-\frac{{\left\|Y-X\beta \right\|}^{2}}{2\sigma^{2}}\right){\left(\sigma^{2}\right)}^{-p/2}r^{p/2}{\left|\Lambda \right|}^{1/2}\exp\left(-\frac{r\beta D^{-1}\beta +r\beta^{T}L\beta }{2\sigma^{2}}\right){\left|\Lambda \right|}^{-1/2}\frac{\lambda^{2}}{2}\exp\left(-\frac{\lambda^{2}}{2}\tau^{2}\right)p\left(r\right)p\left(\sigma^{2}\right)p\left(\lambda \right). \end{array}$$

Integrating out *τ*^2^, we have

(10) $$\begin{array}{c} p\left(\beta ,\lambda ,\sigma^{2},r\;|\;X,Y\right)=\int p\left(\beta ,\lambda ,\sigma^{2},\tau^{2},r\;|\;X,Y\right)p\left(\tau^{2}\right)d\tau^{2}\propto \int_{0}^{\infty }{\left(\sigma^{2}\right)}^{-n/3}\exp\left(-\frac{{\left\|Y-X\beta \right\|}^{2}}{2\sigma^{2}}\right){\left(\sigma^{2}\right)}^{-p/2}r^{p/2}{\left|\Lambda \right|}^{1/2}\exp\left(-\frac{r\beta D^{-1}\beta +r\beta^{T}L\beta }{2\sigma^{2}}\right){\left|\Lambda \right|}^{-2/2}\frac{\lambda^{2}}{2}\exp\left(-\frac{\lambda^{2}}{2}\tau^{2}\right)p\left(r\right)p\left(\sigma^{2}\right)p\left(\lambda \right)d\tau^{2}\propto \int_{0}^{\infty }\exp\left(-\frac{{\left\|Y-X\beta \right\|}^{2}+r\beta^{T}L\beta }{2\sigma^{2}}\right)\exp\left(-\frac{r\beta D^{-1}\beta }{2\sigma^{2}}\right)\frac{\lambda^{2}}{2}\exp\left(-\frac{\lambda^{2}}{2}\tau^{2}\right)d\tau^{2}. \end{array}$$

Applying the fact as follows to the above equation:

(11) $$\begin{array}{c} \frac{a}{2}\exp\left(-a\;|\;z\;|\;\right)=\int_{0}^{\infty }\frac{1}{\sqrt{2\pi s}}\exp\left(-\frac{z^{2}}{2s}\right)\frac{a^{2}}{2}\exp\left(-\frac{a^{2}s}{2}\right)ds,a>0, \end{array}$$

we have

(12) $$\begin{array}{c} p\left(\beta ,\lambda ,\sigma^{2},r\;|\;X,Y\right)\propto \int_{0}^{\infty }\exp\left(-\frac{{\left\|Y-X\beta \right\|}^{2}+r\beta^{T}L\beta }{2\sigma^{2}}\right)\exp\left(-\frac{r\beta D^{-1}\beta }{2\sigma^{2}}\right)\frac{\lambda^{2}}{2}\exp\left(-\frac{\lambda^{2}}{2}\tau^{2}\right)d\tau^{2}=\exp\left(-\frac{{\left\|Y-X\beta \right\|}^{2}+r\lambda \;|\;\beta \;|\;+r\beta^{T}L\beta }{2\sigma^{2}}\right). \end{array}$$

Thus, maximizing the posterior distribution is equivalent to minimizing the following equation:

(13) $$\begin{array}{c} L\left(r,\lambda ,\beta \right)={\left(y-X\beta \right)}^{T}\left(y-X\beta \right)+r\lambda {\left|\beta \right|}_{1}+{\lambda \beta }^{T}L\beta , \end{array}$$

which has the same regularization term as the method proposed in [19].

We assign the prior distribution for *σ*^2^ as follows:

(14) $$\begin{array}{c} \sigma^{2}∼\text{Inverse Gamma}\left(a,b\right). \end{array}$$

And we assign the following prior for the hyperparameters *r* and *λ*:

(15) $$\begin{array}{c} \begin{array}{c} r∼\text{Gamma}\left(c,d\right),\\ \lambda ∼\text{Gamma}\left(e,f\right). \end{array} \end{array}$$

Then, the hierarchical Bayesian model is

(16) $$\begin{array}{c} \begin{array}{c} Y\;|\;X,\beta ,\sigma^{2}∼N_{n}\left(X\beta ,\sigma^{2}I_{n}\right),\\ \beta \;|\;\sigma^{2},\tau^{2},r∼N_{p}\left(0,\frac{\sigma^{2}}{r}\Lambda^{-1}\right),\\ \tau^{2}\;|\;\lambda ∼{\left|\Lambda \right|}^{-1/2}\frac{\lambda^{2}}{2}\exp\left(-\frac{\lambda^{2}}{2}\tau^{2}\right),\\ \sigma^{2}∼\text{Inverse Gamma}\left(a,b\right),\\ r∼\text{Gamma}\left(c,d\right),\\ \lambda ∼\text{Gamma}\left(e,f\right). \end{array} \end{array}$$

### 2.2. Gibbs Sampling Method

The likelihood is

(17) $$\begin{array}{c} p\left(y\;|\;X,\beta ,\sigma^{2}\right)\propto {\left(\sigma^{2}\right)}^{-n/2}\exp\left(-\frac{{\left(Y-X\beta \right)}^{T}\left(Y-X\beta \right)}{2\sigma^{2}}\right). \end{array}$$

According to the above hierarchical model and the likelihood, the joint posterior distribution on data is

(18) $$\begin{array}{c} p\left(\beta ,\sigma^{2},\tau^{2},\lambda^{2},r\;|\;Y,X\right)\propto {\left(\sigma^{2}\right)}^{-n/2}\exp\left(-\frac{{\left(y-X\beta \right)}^{T}\left(y-X\beta \right)}{2\sigma^{2}}\right){\left(\sigma^{2}\right)}^{-p/2}r^{p/2}{\left|\Lambda \right|}^{1/2}\exp\left(-\frac{r\beta^{T}\Lambda \beta }{2\sigma^{2}}\right){\left|\Lambda \right|}^{-1/2}\overset{p}{\underset{j=1}{\prod }}\frac{\lambda^{2}}{2}\exp\left(-\frac{\lambda^{2}}{2}\tau_{j}^{2}\right){\left(\sigma^{2}\right)}^{-a}\exp\left(-\frac{b}{\sigma^{2}}\right)r^{-c}\exp\left(-dr\right){\left(\lambda^{2}\right)}^{-e}\exp\left(-f\lambda^{2}\right). \end{array}$$

Due to the fact that all the prior distributions are conjugated, the full conditional posterior distributions for the parameters have closed forms.

(19) $$\begin{array}{c} p\left(\beta ,\;|\;\sigma^{2},\tau^{2},r,Y,X\right)\propto \exp\left(-\frac{{\left(Y-X\beta \right)}^{T}\left(Y-X\beta \right)}{2\sigma^{2}}\right)\exp\left(-\frac{r\beta \Lambda \beta }{2\sigma^{2}}\right)\propto \exp\left(-\frac{\left(X^{\prime }X+r\Lambda \right)\beta^{2}-2YX\beta }{2\sigma^{2}}\right). \end{array}$$

Let *μ* = (*X*′*X* + *rΛ*)^−1^*X*′*Y*, *Σ* = *σ*^2^(*X*′*X* + *rΛ*)^−1^ , we have

(20) $$\begin{array}{c} \beta \;|\;\sigma^{2},\tau^{2},r,X,Y∼N_{p}\left(\mu ,\Sigma \right), \end{array}$$

(21) $$\begin{array}{c} p\left(\sigma^{2}\;|\;\beta ,\tau^{2},r,Y,X\right)\propto {\left(\sigma^{2}\right)}^{-n/2}\exp\left(-\frac{{\left(y-X\beta \right)}^{T}\left(y-X\beta \right)}{2\sigma^{2}}\right){\left(\sigma^{2}\right)}^{-p/2}\exp\left(-\frac{r\beta^{T}\Lambda \beta }{2\sigma^{2}}\right){\left(\sigma^{2}\right)}^{-a}\exp\left(-\frac{b}{\sigma^{2}}\right)\propto {\left(\sigma^{2}\right)}^{-n+p/2-a}\exp\left(\left(-\frac{{\left(y-X\beta \right)}^{T}\left(y-X\beta \right)+r\beta^{T}\Lambda \beta }{2}+b\right)\frac{1}{\sigma^{2}}\right), \end{array}$$

(22) $$\begin{array}{c} \sigma^{2}\;|\;\beta ,\tau^{2},r,Y,X∼\text{Inverse Gamma}\left(\frac{n+p}{2}+a,\frac{{\left(y-X\beta \right)}^{T}\left(y-X\beta \right)+r\beta^{T}\Lambda \beta }{2}+b\right), \end{array}$$

(23) $$\begin{array}{c} p\left(\tau^{2}\;|\;\beta ,\sigma^{2},\lambda^{2},r\right)\propto \exp\left(-\frac{r\beta^{T}\Lambda \beta }{2\sigma^{2}}\right)\frac{\lambda^{2}}{2}\exp\left(-\frac{\lambda^{2}}{2}\tau^{2}\right). \end{array}$$

This implies that *τ*^2^ follows a generalized inverse Gaussian distribution:

(24) $$\begin{array}{c} \tau_{j}^{2}\;|\;\beta ,r,\sigma^{2},\lambda^{2}∼\text{GIG}\left(\frac{1}{2},\lambda^{2},\frac{r\beta_{j}^{2}}{\sigma^{2}}\right),\;j=1,2,\cdots ,p, \end{array}$$

(25) $$\begin{array}{c} p\left(r\;|\;\beta ,\sigma^{2},\tau^{2}\right)\propto r^{p/2}\exp\left(-\frac{r\beta^{T}\Lambda \beta }{2\sigma^{2}}\right)r^{c}\exp\left(-dr\right)\propto r^{{}^{p/2}+c}\exp\left(-\left(\frac{\beta^{T}\Lambda \beta }{2\sigma^{2}}+d\right)r\right), \end{array}$$

(26) $$\begin{array}{c} r\;|\;\sigma^{2},\beta ,\tau^{2}∼\text{Gamma}\left(\frac{p}{2}+c,\frac{\beta^{T}\Lambda \beta }{2\sigma^{2}}+b\right), \end{array}$$

(27) $$\begin{array}{c} p\left(\lambda^{2}\;|\;\tau^{2}\right)\propto \overset{p}{\underset{j=1}{\prod }}\frac{\lambda^{2}}{2}\exp\left(-\frac{\lambda^{2}}{2}\tau_{j}^{2}\right){\left(\lambda^{2}\right)}^{e}\exp\left(-f\lambda^{2}\right)\propto {\left(\lambda^{2}\right)}^{p+e}\exp\left(-\left(\frac{1}{2}\overset{p}{\underset{j=1}{\sum }}\tau_{j}^{2}+f\right)\lambda^{2}\right), \end{array}$$

(28) $$\begin{array}{c} \lambda^{2}\;|\;\tau^{2}∼\text{Gamma}\left(p+e,\frac{1}{2}\overset{p}{\underset{j=1}{\sum }}\tau_{j}^{2}+f\right). \end{array}$$

The Gibbs sampling scheme iterates as follows:

1. Update *β* by sampling from (20)
2. Update *σ*^2^ by sampling form (22)
3. Update *τ*^2^ by sampling from (24)
4. Update *r* by sampling from (26)
5. Update *λ* by sampling from (28)

### 2.3. The Binary Response Case

Binary data such as absence or presence or different types of a disease are often used as response variables in gene selection problems. To perform binary classification, we use probit regression using auxiliary variables. Then, the model can be represented as follows:

(29) $$\begin{array}{c} P\left(y_{i}=1\right)=X_{i}\beta , \end{array}$$

where *X*_*i*_ is the *i*th sample and *P*(*y*_*i*_ = 1) is the probability of *y*_*i*_ = 1. Here, latent variables *Z* = (*z*_1_, *z*_2_, ⋯, *z*_*n*_) are defined as

(30) $$\begin{array}{c} z_{i}=X_{i}\beta +\varepsilon ,\varepsilon ∼N_{n}\left(0,\sigma^{2}I_{n}\right). \end{array}$$

Then, the full conditional posterior distribution for each *z*_*i*_ is truncated normal:

(31) $$\begin{array}{c} z_{i}\;|\;\beta ,X_{i},y_{i}∼\left\{\begin{array}{c} N\left(X_{i}\beta ,\sigma^{2}\right)I\left(z_{i}>0\right),\;y_{i}=1,\\ N\left(X_{i}\beta ,\sigma^{2}\right)I\left(z_{i}\leq 0\right),\;\text{otherwise}. \end{array}\right. \end{array}$$

And *Z* follows a multivariate truncated normal distribution:

(32) $$\begin{array}{c} p\left(Z\;|\;\beta ,\sigma^{2},X,Y\right)\propto N_{n}\left(X\beta ,\sigma^{2}I_{n}\right)\overset{n}{\underset{i=1}{\prod }}I\left(A_{i}\right), \end{array}$$

(33) $$\begin{array}{c} A_{i}=\left\{\begin{array}{c} \left\{Z_{i}\;|\;Z_{i}>0\right\},\left(Y_{i}=1\right),\\ \left\{Z_{i}\;|\;Z_{i}\leq 0\right\},\left(Y_{i}=0\right). \end{array}\right. \end{array}$$

Sampling from this distribution directly is difficult. We use the method proposed in [26] to sample this latent variable.

Then, the hierarchical Bayesian model is

(34) $$\begin{array}{c} \begin{array}{c} Z\;|\;X,Y,\beta ,\sigma^{2}∼N_{n}\left(X\beta ,\sigma^{2}I_{n}\right)\overset{n}{\underset{i=1}{\prod }}I\left(A_{i}\right),\\ \beta \;|\;\sigma^{2},\tau^{2},r∼N_{p}\left(0,\frac{\sigma^{2}}{r}\Lambda^{-1}\right),\\ \tau^{2}\;|\;\lambda ∼{\left|\Lambda \right|}^{-1/2}\frac{\lambda^{2}}{2}\exp\left(-\frac{\lambda^{2}}{2}\tau^{2}\right),\\ \sigma^{2}∼\text{Inverse Gamma}\left(a,b\right),\\ r∼\text{Gamma}\left(c,d\right),\\ \lambda ∼\text{Gamma}\left(e,f\right). \end{array} \end{array}$$

To derive the Gibbs sampling scheme, we only need to replace *Y* with *Z* in the Gibbs sampling scheme defined in Section 2.2. And the latent variables *Z* are sampled from (32).

## 3. Results

### 3.1. Datasets and Preprocessing

To demonstrate the effectiveness of our methods, a regression microarray dataset and 5 real-life binary classification microarray datasets were tested in this paper, which are described as follows. The pathway information was obtained from the KEGG database.

A breast cancer dataset was used to predict the survival time of patients [27]. We used gene expression profiles of 76 patients. Each patient was measured with 24481 probes. 3592 genes were found in the KEGG database from this dataset. We used the logarithm of survival times of patients as the response variable in this dataset.

The other 5 binary classification microarray datasets are shown in Table 1. No. genes mean the genes we found both existing in the microarray dataset and KEGG pathway database.

Lastly, the gene expression values were normalized; thus, its mean and standard deviation are 0 and 1.

### 3.2. Parameter Settings

In the procedure of Bayesian network-constrained regularization, we recommend small values for *a*, *b*, *c*, *d*, *e*, *f* in (16) and we set these values to 0.01 in our experiments. The Gibbs sampling iteration was conducted 6000 times, and we chose the second half of the samples to estimate the regression parameters. The posterior estimates of all parameters were obtained through the posterior averages of the chains. For the classification problem, the classifiers were built by a support vector machine (SVM). In this paper, we used the radial basic function as the kernel function in SVM. And the regularization parameter and the kernel width parameter were optimized by a grid search approach. We used Libsvm [32] to model the SVM.

### 3.3. Results and Analysis

In this section, we will describe the results on 6 microarray gene expression datasets (Table 1) to evaluate the performance of the proposed method. Our method was compared with the other three Bayesian regularized regression methods, including Bayesian Lasso, Bayesian Elastic Net, and Bayesian Fused Lasso. A comprehensive review of these methods can be found in [23]. When *L* = *I*, which means we know nothing about the pathway structure, the Bayesian network-constrained regularization is equivalent to Bayesian Elastic Net. And when *L* = *O*, our method is equivalent to Bayesian Lasso. These three methods can also be extended to perform binary classification through an auxiliary variable. We also used Gibbs sampling to perform parameter estimation. Previous review [23] also shows that these three Bayesian methods' performances are similar to and in some cases better than the frequentist methods. Prediction mean square error was used to evaluate the performance on regression problem. Meanwhile, ACC and AUC were used as the evaluation criteria for binary classification problem. According to previous studies, the number of important genes is probably about 50 [28]; thus, we selected the top 50 genes based on the absolute value of their regression coefficient for the binary classification problem.

Figure 1 shows the performance of all the four methods on the regression microarray dataset. And the classification performances on the five binary classification microarray datasets are summarized in Table 2. In the binary classification datasets, the first three datasets are usually treated as easy classification datasets, while the other two datasets are relatively hard to classify. From Figure 1, we can see that the PMSE of our method is lower than other Bayesian methods. Table 2 also shows that on the four easy binary classification datasets, our method achieves the highest ACC and AUC. In the other two hard classification datasets, our method achieves the highest ACC and AUC on GSE412. Although the AUC of Bayesian Elastic Net is higher than our method on GSE4922, our method achieves the highest ACC. In general, Bayesian network-constrained regularization shows better prediction and classification ability than other three Bayesian methods, which is similar to the results implied by [15]. Since our method can be transferred to Bayesian Lasso or Bayesian Elastic Net when the normalized Laplacian matrix *L* = *O* or *L* = *I*, the results also show that pathway information indeed contributes to the accuracy of the gene selection.

Consistent with previous studies [33, 34], all the Bayesian regularization regression methods could classify Leukemia, DLBCL, Prostate, and GSE412 dataset accurately. However, the performances of all the methods were poor on GSE 4922 dataset. Therefore, we demonstrate the effectiveness of our method by selecting the top 18 genes which make the prediction accuracy to achieve the highest value and most of those genes are associated with breast cancer (Table 3).

## 4. Conclusion

In this paper, we propose a Bayesian approach to perform gene selection, which can incorporate the pathway information as prior biological knowledge through network-constrained regularization to improve the accuracy of gene selection. All the prior distributions we propose are strictly conjugated; thus, all the conditional posteriors of the model are available in closed form. An auxiliary variable is also introduced to extend the regression model to perform binary classification. An efficient Gibbs sampling method is used to estimate regression coefficients and tune parameters simultaneously, which can perform feature filter feasible for high dimensional microarray datasets. The performance of the proposed method is demonstrated by applying it to a regression microarray dataset and five binary classification microarray datasets. The results show that compared with Bayesian Lasso, Bayesian Elastic Net, and Bayesian Fused Lasso, our method performs better both in prediction and classification. And the pathway information indeed improves the accuracy of gene selection.

## Figures and Tables

**Figure 1:** PMSE performance on regression microarray dataset.

**Table 1:** Binary classification microarray datasets used.

Dataset name	No. genes	Samples	P/N	References
Leukemia	1883	72	47/25	[28]
DLBCL	2427	77	58/24	[29]
Prostate	3238	102	50/52	[30]
GSE412	3234	108	60/48	[31]
GSE4922	4476	204	70/134	[26]

**Table 2:** Comparison of results of 4 Bayesian methods.

Dataset	Methods	AUC	ACC
Leukemia	BEN	0.9955	0.9600
	BFused	1	0.9733
	BLasso	1	0.9447
	BNR	1	0.9733
DLBCL	BEN	0.9674	0.9223
	BFused	0.9674	0.9223
	BLasso	0.9485	0.9223
	BNR	0.9958	0.9482
Prostate	BEN	0.9784	0.9414
	BFused	0.9655	0.9314
	BLasso	0.9784	0.9419
	BNR	0.9900	0.9510
GSE412	BEN	0.9428	0.8498
	BFused	0.9046	0.8619
	BLasso	0.9541	0.8792
	BNR	0.9637	0.9074
GSE4922	BEN	0.6274	0.6666
	BFused	0.6028	0.6523
	BLasso	0.6132	0.6860
	BNR	0.6132	0.6860

**Table 3:** Description of top 18 genes of GSE4922.

Gene symbol	Description	Reference
SYCP3∗	Synaptonemal complex protein 3	[35]
CDKN2A∗	Cyclin dependent kinase inhibitor 2A	[36]
PLB1∗ CTNNBIP1∗	Phospholipase B1 Catenin beta-interacting protein 1	[37] [38]
GBE1∗	1,4-Alpha-glucan-branching enzyme 1	[39]
SMURF1∗	SMAD-specific E3 ubiquitin protein ligase 1	[40]
NR1H4	Nuclear receptor subfamily 1 group H member 4	/
PDE11A	Phosphodiesterase 11A	/
UGT1A1∗	UDP glucuronosyltransferase family 1 member A1	[41]
FGF19∗	Fibroblast growth factor 19	[42]
OR51B4∗	Olfactory receptor family 51 subfamily B member 4	[43]
RAB7A∗	RAB7A, member RAS oncogene family	[44]
SDHD∗	Succinate dehydrogenase complex subunit D	[45]
IFNA8	Interferon alpha 8	/
VANGL2∗	VANGL planar cell polarity protein 2	[46]
UMPS	Uridine monophosphate synthetase	/
CASP3	Caspase 3	[47]
SUFU	SUFU negative regulator of hedgehog signaling	[48]

^∗^The gene was reported as an oncogene in previous literatures.

## Data Availability

The breast cancer dataset could be obtained from the R package breast cancer NKI. Leukemia, DLBCL, and Prostate datasets are available on the website http://portals.broadinstitute.org/cgi-bin/cancer/. GSE412 and GSE4922 datasets are available in the GEO of NCBI under accession GSE412 and GSE4922.
